The article "Classification of Alzheimer's Disease Using Gaussian-Based Bayesian Parameter Optimization for Deep Convolutional LSTM Network" was retracted in 2023. Reasons: signs of a paper mill; compromised peer review; unreliable results or conclusions.

# Classification of Alzheimer's Disease Using Gaussian-Based Bayesian Parameter Optimization for Deep Convolutional LSTM Network

**DOI:** 10.1155/2021/4186666

**Published:** 2021-10-04

**Authors:** Monika Sethi, Sachin Ahuja, Shalli Rani, Puneet Bawa, Atef Zaguia

**Affiliations:** ^1^Chitkara University Institute of Engineering and Technology, Chitkara University, Punjab 140401, India; ^2^Centre of Excellence for Speech and Multimodal Laboratory, Chitkara University Institute of Engineering & Technology, Chitkara University, Punjab, India; ^3^Department of Computer Science, College of Computers and Information Technology, Taif University, P.O. Box 11099, Taif 21944, Saudi Arabia

## Abstract

Alzheimer's disease (AD) is one of the most important causes of mortality in elderly people, and it is often challenging to use traditional manual procedures when diagnosing a disease in the early stages. The successful implementation of machine learning (ML) techniques has also shown their effectiveness and its reliability as one of the better options for an early diagnosis of AD. But the heterogeneous dimensions and composition of the disease data have undoubtedly made diagnostics more difficult, needing a sufficient model choice to overcome the difficulty. Therefore, in this paper, four different 2D and 3D convolutional neural network (CNN) frameworks based on Bayesian search optimization are proposed to develop an optimized deep learning model to predict the early onset of AD binary and ternary classification on magnetic resonance imaging (MRI) scans. Moreover, certain hyperparameters such as learning rate, optimizers, and hidden units are to be set and adjusted for the performance boosting of the deep learning model. Bayesian optimization enables to leverage advantage throughout the experiments: A persistent hyperparameter space testing provides not only the output but also about the nearest conclusions. In this way, the series of experiments needed to explore space can be substantially reduced. Finally, alongside the use of Bayesian approaches, long short-term memory (LSTM) through the process of augmentation has resulted in finding the better settings of the model that too in less iterations with an relative improvement (RI) of 7.03%, 12.19%, 10.80%, and 11.99% over the four systems optimized with manual hyperparameters tuning such that hyperparameters that look more appealing from past data as well as the conventional techniques of manual selection.

## 1. Introduction

AD permanent neurological condition occurs rapidly and progresses continually, marked by cognitive dysfunction [1], modifications in behaviour [2], language disorientation, and delusions [3, 4]. AD is perhaps the most predominant cause of dementia and the second biggest cause of mortality in the United States [5]. The major research topic by the Association of Alzheimer [6] indicates the existence of about 5 million US people with AD. One new case of AD is predicted to arrive every 30 seconds, and the estimated number is expected to reach at about 14 million by 2050. The instantaneous and haphazard costs of AD-identified medical treatment across the regions of the United States and Europe are alone estimated at almost $500 billion annually [7]. The diagnosis of AD relies on clinical assessment and prolongation of patients alongside their family consultation [8, 9]. In any case, ‘a well ground truth' finding of AD must be formed utilizing postmortem examination, which is not clinically relevant. Patients need some other basis to confirm AD without ground truth information. Such type of criteria could improve our comprehension of AD and make it easier for live patients to identify those [10]. There is no well-known cure for AD, yet a very few treatments allow it to postpone its course [11]. Therefore, early detection of MCI subjects at higher risk for transitioning to AD is as significant as highlighted in a notable discourse conveyed by German neuropathologist and psychiatrist Dr. Alois Alzheimer in which he clarified interestingly the sort of dementia, which was subsequently named with his name itself as Alzheimer's disease [12]. He introduced a 51-year-old woman from Frankfurt who had passed on because of extreme psychological instability [13]. He analysed her mind and discovered amyloidal plaques and a heap of strands [14, 15] that were brought about by unusual protein testimony in and around the neuron cells. Since healthier neurons in the cerebrums stop working appropriately, suddenly, they start losing out their associations with a few other neurons and consequently die [16]. Thus, the volume of the hippocampus and cerebral cortex is diminished while the cerebral ventricles are broadened further influencing the bits of the speculative mind, long-term memory, and handling the data coming out from five senses [17]. However, the severity of all these disruptions in the brain depends on the extent of the disease such as extreme shrinkage of the cerebral cortex and hippocampus and the expansion of the ventricles could be seen straight ahead in brain imaging during the later stage of the disease [18]. In a like manner, sufferers at the earliest stage of AD are alluded to as MCI although not all MCI cases may grow AD [19]. MCI is a transitional stage [20, 21] from healthy to AD, during which the individual has mild behavioural changes that really are noticeable to the individuals who are affected as well as to the members of the family. In such cases, the transitional duration tends to differ from 6 to 36 months, though 12-18 months are common [22]. Thus, MCI sufferers are then categorized as MCI converters and MCI nonconverters. However, the exact causes of AD are yet not well understood to healthcare professionals and no proven medicines or therapies have even been confirmed to prevent or reverse the progression of AD [23].

The article "Classification of Alzheimer's Disease Using Gaussian-Based Bayesian Parameter Optimization for Deep Convolutional LSTM Network" was retracted in 2023. Reasons: signs of a paper mill; compromised peer review; unreliable results or conclusions.

Fortunately, early diagnosis of AD offers sufferers prior knowledge about the seriousness and encourages them to take appropriate steps, e.g. dietary modifications and medication, that may significantly improve their memory and their quality of life as well [24]. Diagnosing AD accurately at an initial level is, thus, of huge importance. To support AD diagnosis, many past studies used images from numerous noninvasive neuroimaging biomarkers such as structural, functional, and molecular imaging. Structural imaging such as structural MRI (sMRI) and computed tomography reveals the significant amount of information regarding the structural changes (position, volume, and shape) inside the brain [16]. Functional imaging such as functional MRI and positron emission tomography (PET) are often used to illustrate the working of cells in different brain areas by demonstrating the sugar and oxygen level usage by them. Molecular imaging such as single-photon emission computed tomography is used to identify the chemical and cellular modifications that are related to particular disease with radiotracers. MRI or the combination of MRI and PET [25, 26] are often used to diagnose AD. Due to the heterogeneous nature of these imaging data, it would obviously be tedious to compare, analyse, and visualize it [27]. The sMRI is one of the most common techniques, as it can provide a strong resolution between the subcortical brain tissues and the grey matter area. In recent years, there has been a major transition further towards nonlinear methodologies, despite some initial success of support vector machines (SVM) and linear classifiers [1]. The advent of utilization of such scans, in particular, has widened the scope of automated diagnosis and detection of AD through the process of image recognition. In development, however, these practices have changed. To extricate the features from MRI and PET neuroimaging data in [28], a deep Boltzmann machine has been utilized and later the part of acquisition has been implemented baked on the cognitive scores and cerebrospinal fluid (CSF) in addition to such classification of MRI and PET neuroimaging data.

The acquisition of such scans is done with lesser amount of energy resulting in the low contrast and bad quality of an image with essential need of human intervention. Thus, computer-aided diagnostic systems have been developed which play a pivotal role in improving the quality of medical images highlighting the conspicuous parts more effectively [29]. Likewise, the use for the family of ML techniques has increased exponentially over the past decades with an effort of diagnosing and classifying cognitive normal (CN), AD, and mild cognitive impairment (MCI) subjects. Furthermore, many ML and DL techniques for early detection of AD have been evaluated using the above discussed neuroimaging modalities through the process of image detection and recognition. In a like manner, many endeavours have been looked upon by the researchers concerning the parametric optimization of the model with an objective of early diagnosis and detection of the disease. Such type of classifiable models inherits the several steps including the process for extraction and adequate selection of data features corresponding to an input image, thus reducing the dimensions of those selected features, and resulting into the effective performance under such classification. Typically, the classification model utilized for the same involves minimally two steps including the aforementioned feature extraction process and secondly the use of classification algorithms to promote automatic decision support in biomedical fields [30]. However, the extraction of these features involves human experts who typically need a lot of dedication, budget, and time. Moreover, researchers have suggested different automated methods of selecting ML algorithms and/or the hyperparameter values for a given supervised machine-learning problem in order to make ML available to layman users [31]. The aim of these techniques is to rapidly discover an efficient algorithm and/or combination of hyperparametric values within a prespecified resource limit that maximizes the accuracy of the ML problem and dataset. The area below the receiver operating characteristic curve is an example of a precision measure. The limit of resources will normally be determined by time, the number of algorithms and/or hyperparameter combinations checked in the dataset, or by the number of scans conducted over the training data [32]. The user of a ML software tool should use an automated selection method to skip the manual and iterative process of choosing an efficient algorithm and/or combination of labour-intensive hyperparameter values that requires a high level of ML abilities. Lately, with the advancement of DL models' subarea of ML, it is possible to identify even the complex level of features directly from imaging data without much human intervention.

The article "Classification of Alzheimer's Disease Using Gaussian-Based Bayesian Parameter Optimization for Deep Convolutional LSTM Network" was retracted in 2023. Reasons: signs of a paper mill; compromised peer review; unreliable results or conclusions.

In this paper, an effort has been made for early detection of AD with comparisons of modelling efficacy being conducted using the four different systems: considering the ternary classification as (a) AD, MCI, CN, and binary per mutational classification, (b) AD and MCI, (c) CN and MCI, and (d) AD and CN. Through this work, the following contributions considering the use of abovementioned classification systems have been made:

- An optimized new set of models based on Bayesian parameter optimization of the deep learning model for the classification of AD is proposed
- The framework also includes comparative analysis of 2D and 3D convolutional architecture on MRI neuroimaging data
- The combination of Bayesian optimized parameters utilizing long short-term memory (LSTM) through the augmentation process has succeeded in discovering better model settings with minimal iteration and increased performance
- Increased accuracy on adoption before clinical diagnosis to anticipate conversion to Alzheimer's disease

These developed systems further have been comparatively evaluated utilizing multimodel DL approaches. Therefore, Bayesian methods of optimization are very effective at a very high level yet take a little longer for the optimally selecting the next hyperparameters such that the time spent for the choice of hyperparameters in reality is inconsistent with the time spent on the objective function.

The remainder of the paper is organized as follows: Section 2 includes the literature review for various images and model selection techniques with Section 3 detailing the theoretical context of the deep learning models. Further, Section 4 shows the details in the dataset utilization alongside the measurement of cognitive assessment test with the proposed system architecture described in Section 5, and finally, the conclusion for comparative study using a novel algorithm for optimal selection was shown in Section 6.

## 2. Related Work

Different modalities of medical imaging data include computerized tomography scans; sMRI, functional MRI, and diffusion tensor imaging have been used to diagnose AD in various ways using diverse ML algorithms [33–36]. Azari et al. [36] submitted in the early 1990s a new statistical technique for assessing the variations between rCMR_glc_ interdependencies in the individual patterns corresponding to PET data of mild and moderately demented patients. Likewise, the researcher implemented multiple regressions and the process of discriminatory analysis to differentiate patients from controls and also to identify early AD trends correlated with independent memory impairment. In [37], further, the researcher group considered the advancement of clinical instrumentation based on multimodality with the aim of designing current technologies and further explored the potential for devices that incorporate these multimodal techniques. The authors in [38] proposed the first work to use not only the neuroimaging data but also combined the CSF biomarkers also using a kernel combination method to classify AD (or MCI) and healthy control (HC). Particularly, baseline MRI, fluorodeoxyglucose-PET, and CSF data of 52 (HC), 99 (MCI), and 51 (AD) subjects were collected from Alzheimer's disease neuroimaging initiative (ADNI). Only volumetric features from the 93 ROIs were extracted for each MRI or fluorodeoxyglucose-PET neuroimage whereas the original values were utilized as features for CSF biomarkers. To evaluate the classification accuracy, a linear SVM was utilized using 10-fold cross-validation. To classify AD with HC, a polynomial kernel with SVM was proposed in [39] to extricate the features of the MRI neurodata obtained from ADNI using a multiscale fractal technique. However, the definition and extraction of features usually depend upon the manual or semiautomatic outlines of the brain structures that are difficult and susceptible for intra-/interrater variability, computationally challenging, and time-consuming. A methodology was suggested in [40] by extension of neuroimaging data with biological facts; particularly, they included voxel-based PET signal intensities, CSF, MRI volumes, and genetic data. The classification was done using the random forest classifier based on all four different combinations of modalities. As compared to multikernel, classifiers based on SVM achieved a comparable accuracy of 89% for AD/HC and 75% for MCI/HC. In contrast, authors in [41] combined MRI neuroimaging data only with cognitive and age-related data. The authors purposely avoided the use of PET and CSF biomarkers due to their unavailability in comparison to MRI, and likewise, these biomarkers are invasive and potentially painful for the patient. After the data collection, semisupervised SVMs were utilized to classify MCI and AD.

The article "Classification of Alzheimer's Disease Using Gaussian-Based Bayesian Parameter Optimization for Deep Convolutional LSTM Network" was retracted in 2023. Reasons: signs of a paper mill; compromised peer review; unreliable results or conclusions.

The experimental results in [42] have shown that a random search is an effective approach for the selection of the hyperparameters for a given ML algorithm. As compared to a thorough and exhaustive search, the hyperparameter grid is much more efficient. Only a few hyperparameters matter for a particular ML algorithm; others may not have any influence on the model's performance. In [43], researchers defined a methodology for quantifying the significance of various hyperparameters. In another research paper [44], authors implemented an autoselective freeze-thaw strategy for automatic hyperparameter selection with a hypothesis that the model's error rate decays exponentially during the training process. This technique preserves a number of partially completed models, using its estimated final accuracy, at any point in the sequential model-based optimization process, to decide whether to freeze an older model, carry on training a part-finished model, or start training a new model with a different combination of hyperparameter values. This saves additional expense due to the unexceptional, partly completed model of continued training. In a similar way, the authors in [45] developed a technique for automatic selection of the hyperparameters. For various combinations of hyperparameters, the technique stores the experimental results for the previous experiment's results for the model's accuracy. The technique is based on the Gaussian regression process to predict the ranking of various combinations of hyperparameters. In [46], the researcher's group developed two different strategies for the automatic hyperparameter selection process. Benefited from an alternative family of ML techniques, termed DL algorithms, and with the accumulation of clinical data, researchers are now achieving optimal results in multiple areas like computer vision, language processing, speech recognition [47], and the area of medical imaging [48–50]. DL techniques vary from the traditional ML techniques by the fact that they either require no or little preprocessing of images and then can infer the features automatically from the raw imaging data without the human intervention leading to less bias-prone and more purposeful results. Thus, DL models are ideally suited for detecting complex and diffuse neuroanatomical changes. CNN has become popular among DL models. Several CNN variants were used by researchers such as proposed 2D CNN architectures to learn slice-wise features from the MRI images of the ADNI dataset [51]. The sparse autoencoder was trained first on the randomly selected patches of natural images. The learned parameters were then utilized as the filters of the CNN's convolutional layer. In [52], the authors adopted the same strategy; they initially used sparse autoencoder to learn the filters for the first convolution layer of the 3D CNN model on randomly chosen 3D patches of the MRI neuroscans of the ADNI dataset. Similarly, the researchers in [53] suggested a 3D CNN network to predict AD that was pretrained by the 3D convolution autoencoder (3D CAE). The general features were captured by the 3D CAE using CAD dementia MRI dataset; then, for target specific classification, top fully connected layers of 3D CNN were fine-tuned on the ADNI dataset. In [54], cascaded 3D CNN architectures were adopted to learn hierarchical features from PET images. Firstly, to convert the local image into high-level features, several 3D-CNNs were built on various local patches of image and then to classify those features were orchestrated using a deep 3D CNN. Their model achieved a good performance level. Researchers in [55] used the DL model to integrally analyse MRI, genetic, and clinical datasets to categorize subjects into CN, MCI, and AD. Specifically, autoncoders stacked for genetic and clinical data extraction and the 3D-CNN for MRI neuroimaging data have been employed. The results showed that DL models were more successful with respect to performance metrics than those of the shallow models, including SVM and random forest. Furthermore, in [56], the authors introduced a new classification framework to capture the features of the image slices using RNN-GRU. Through the combination of the CNN and RNN, the researcher incorporated the interstitial functions which resulted in promising AUC rates of 95.3% and 83.9%, respectively, for AD vs. normal control (NC) and NC vs. MCI classification. A new paradigm for DL through the use for deeper spatial mapping of a hybrid technique was developed of fully stacked bidirectional (FSBi) and LSTM models was developed in [57]. AUC of 94.82%, 86.36%, and 65.3% in NC vs. AD, NC vs. pMCI, and NC vs. sMCI respectively have resulted from a system of MRI and PET base image acquisition. Another researcher group in [58] adopted Siamese CNN models inspired by the transfer of VGG-16 learning to classify different AD stages. Especially, challenges identified by unbalanced and insufficient data are addressed employing data augmentation techniques on the OASIS dataset. An ensemble network of CNN, RNN, and LSTM using a weighted average approach on the OASIS dataset at first, and then, a bagging technique was applied on individual networks to decrease the variance factor in [59]. Finally, bagged models were combined with the use of ensemble and achieved a high accuracy of 92.22%. Transfer learning VGG architecture-based network on the ADNI dataset to classify 4 different classes AD, NC, and early and late MCI and achieved highest accuracy for AD vs. NC as 98.73% and other remaining classes, on the other hand, have an accuracy rate of over 80% [60].

The article "Classification of Alzheimer's Disease Using Gaussian-Based Bayesian Parameter Optimization for Deep Convolutional LSTM Network" was retracted in 2023. Reasons: signs of a paper mill; compromised peer review; unreliable results or conclusions.

## 3. Theoretical Background

### 3.1. Convolution Neural Network

ConvNet or alluded to as CNN is a conventional algorithm utilized in DL with image as an input based on the significance of attributes including learnable weights, tendencies, and biases added to them alongside the differentiations existing between them. However, in correlation to other classification algorithms, the proportion of preprocessing required by a CNN is significantly less. Although primitive methods require hand-engineering of filters, yet architecture of CNN is well suitable to become familiar with these qualities reliant on enough data training. Likewise, the network is well able to capture the spatial and temporal dependencies in an MRI scans both if there should arise an occurrence of 3D and 2D relating to the clinical imaging through the cycle of reduction and viable optimization parameters [61].

The important aspect in architecture includes the definition of the convolution product which is being done after implication of basic operations including padding and stride. The convolution products are therefore evaluated as a two-dimensional matrix with the end objective that each element is related to the sum of the element of the cube (filter) and the sub cube of the image is given as

(1) $$\begin{array}{c} \text{conv}{\left(I,S\right)}_{a,b}=\overset{n_{x}}{\underset{i=1}{\sum }}\overset{n_{y}}{\underset{j=1}{\sum }}\overset{n_{c}}{\underset{k=1}{\sum }}I_{a+i-1,b+j-1,k}.S_{i,j,k}, \end{array}$$

and the dimensions for such representation are being noted as in

(2) $$\begin{array}{c} \dim\left(\text{conv}\left(I,S\right)\right)=\left\{\begin{array}{cc} \left\lfloor \frac{\left(n_{X}+2p-f\right)}{n_{s}}+1\right\rfloor ,\left\lfloor \frac{\left(n_{y}+2p-f\right)}{n_{s}}+1\right\rfloor , & n_{s}>0,\\ n_{X}+2p-f,n_{y}+2p-f, & n_{s}=0, \end{array}\right. \end{array}$$

where ⌊*x*⌋ is the floor function of *x*, *n*_*x*_ is the height of the image, *n*_*y*_ is the width of the image, *n*_*c*_ is the number of channels, and *p* is for padding factor of convolution through consideration of the filter which is to be squared with an odd dimension being denoted as *f* allowing each pixel to be centred in the filter and consideration of all the elements around the input image dataset. Furthermore, filter slides without knowing about parameters after a certain step and pooling function is applied on the selected elements as in

(3) $$\begin{array}{c} \dim\left(\text{pool}\left(I,S\right)\right)=\left\{\begin{array}{cc} \left\lfloor \frac{\left(n_{X}+2p-f\right)}{n_{s}}+1\right\rfloor ,\left\lfloor \frac{\left(n_{y}+2p-f\right)}{n_{s}}+1\right\rfloor ,n_{c}, & n_{s}>0,\\ \left(n_{X}+2p-f,n_{y}+2p-f,n_{c}\right), & n_{s}=0. \end{array}\right. \end{array}$$

Finally, there are repetitions of such convolutions followed by activation functions with definition of the pooling in the principal step as detailed in Equation (3) and repeat this process several times. This enables the extracted features of an input image to be supplied to a neural network with fully connected layers and activated functions periodically.

The article "Classification of Alzheimer's Disease Using Gaussian-Based Bayesian Parameter Optimization for Deep Convolutional LSTM Network" was retracted in 2023. Reasons: signs of a paper mill; compromised peer review; unreliable results or conclusions.

### 3.2. Long Short-Term Memory

CNN is well structured to accommodate a single image and to transform it into a vector representation. RNN was used to detect image as per the factor time, but in some instances, it was found unreliable in practice because of gradient explosion across long-term windows during the back propagation phase of gradients in an image [62].

The LSTM technique is then used in order to enhance the model efficiency, which can help eliminate the above problem by replacing hidden units by memory cells. This multilayer operation is called the time distributed layer, for internal state building and weight modifications, typically done via back propagation through time in the internal vector representation sequence as done in CNN. This means that the addition of these layers consequently results in several applications of the same layer or layer and a series of “image interpretations” or “image features” to operate on an LSTM architect with

- block input  (*b*_*g*_) in

(4) $$\begin{array}{c} b_{g}=\tanh\left(W_{b}*X_{g}+U_{b}*{\text{out}}_{g-1}+d_{b}\right) \end{array}$$

(ii) input gate (*i*_*g*_) in

(5) $$\begin{array}{c} i_{g}=\sigma \left(W_{i}*X_{g}+U_{i}*{\text{out}}_{g-1}+d_{i}\right. \end{array}$$

(iii) forget gate (*f*_*g*_) in

(6) $$\begin{array}{c} f_{g}=\sigma \left(W_{f}*X_{g}+U_{f}*{\text{out}}_{g-1}+d_{f}\right. \end{array}$$

(iv) memory state  (*m*_*g*_) in

(7) $$\begin{array}{c} m_{g}=i_{g}⊙Z_{g}+f_{g}⊙m_{g-1} \end{array}$$

(v) output gate (*O*_*g*_) in

(8) $$\begin{array}{c} O_{g}=\sigma \left(W_{o}*X_{g}+U_{b}*{\text{out}}_{g-1}+d_{o}\right) \end{array}$$

(vi) and hidden state  (*h*_*g*_) in

(9) $$\begin{array}{c} h_{g}=O_{g}⊙\tanh\left(C_{g}\right) \end{array}$$

## 4. Experimental Setup

### 4.1. Dataset Acquisition and Processing

In order to generate predictive forecasts of potential disease growth for individual patients, the paper is aimed at efficiently improving the classification system by training a deep convolution LSTM neural network on MRI-based 3D and 2D patients' neuroimages. In this work, we used the simple and follow-up visits to ADNI T1-MRI as this modality have numerous images available on ADNI. The data collection documentation is accessible on the website of the ADNI (ADNI: http://adni.loni.usc.edu/) [63], headed by principal investigator Michael W. Weiner, MD. It was established in 2003 as a public-private collaboration with the purpose of identifying more sensitive and effective methodologies for diagnosing whether early AD as well as the development of MCI alongside marking the prognosis through the use of biological markers, clinical and neuropsychological tests.  Figure 1 illustrates a few samples of brain MRI images obtained from the ADNI dataset.

The article "Classification of Alzheimer's Disease Using Gaussian-Based Bayesian Parameter Optimization for Deep Convolutional LSTM Network" was retracted in 2023. Reasons: signs of a paper mill; compromised peer review; unreliable results or conclusions.

Next, the utilization for the total number of sMRI structural scans (*n* = 365) in the Neuroimaging Informatics Technology Initiative (NiFti) format for the three different subjects: CN (*n* = 203), AD(*n* = 109), and MCI (*n* = 53) as baseline has been experimented and then further transformed 3D into 2D paradigm (.png extension) through the process as defined in Algorithm 1. Only the middle slices were considered, and the images at the boundaries were discarded keeping in view that those do not contain any useful information. After the exclusion, the utilization through the division of training and testing with the ratio of 90% and 10% concerning each cohort, CN, MCI, and AD for the training and testing datasets, respectively, has been made for initial development of the baseline system. Considering the same, total number of 183 subjects having a healthy brain (CN), 98 subjects diagnosed with AD, and 47 subjects having MCI were taken into account as the training set, whereas remaining 20 subjects for CN, 11 having AD, and 6 having MCI have been considered for the validation process against the training set. Finally, the individual training of 2D and 3D MRI neuroimages has been performed based on the two dataset classification organizations of the dataset: (1) binary and (2) ternary, resulting as an effective prognostic classification and prediction of the diseases from three sets: CN, MCI, and AD.

Generally, the clinical dementia rating (CDR) is utilized in classification of AD. The CDR ratings vary between 0 and 3, while 5 stages of CDR are 0, 0.5, 1, 2, and 3. For healthy controls, CDR is 0 only. On the other hand, the case is referred to as AD if CDR values are higher than 0.5 or either 1, 2, or 3. For the visualization CDR factor, as shown in Figure 2, 97% of the CN cohorts have CDR scores between 0 and 0.5 and 53% subjects suffering from AD have CDR score lying between 0.6 and 1. More than 50% patients suffering from MCI have a CDR score between 0 and 0.5, and 30% victims have scores between 0.6 and 1 and rest have 1.1 to 3.

### 4.2. Demographic Information

Table 1 illustrates the demographic information along with the age and CDR scores. The subjects chosen were between 56 and 95 years old, and ranges are almost identical for separate subjects. Male and female ratios in AD/MCI subjects are identical while male and female proportions in CN subjects are lower. The average CDR score were calculated for each cohort (CN, MCI, and AD).

The article "Classification of Alzheimer's Disease Using Gaussian-Based Bayesian Parameter Optimization for Deep Convolutional LSTM Network" was retracted in 2023. Reasons: signs of a paper mill; compromised peer review; unreliable results or conclusions.

### 4.3. Dataset Augmentation

In order to improve the performance of the model, further, the technique of data augmentation through rotation was applied on the training set as detailed in Algorithm 2. For each image of the training dataset, rotation transformation using angles of 180 and 270 degrees was performed on the basis such that the features corresponding to the scans of AD/MCI/CN are invariant/insensitive to rotation. For each image, in the first-round angle 180 degree was given for each image of each class, and in the second round, a 270-degree angle was inputted to rotate the images for each class resulting in two types of training datasets were obtained:

- 180-degree augmented training set with number of subjects (CN: 406, MCI: 106, and AD: 218)
- 270-degree augmented training set with number of subjects (CN: 406, MCI: 106, and AD: 218)

Finally, the performance analysis for both abovementioned augmented datasets has been performed validated against the same testing set as detailed for the use in the baseline system.

## 5. System Architecture

For the development of the baseline classification model, we employed 2D CNN and 3D CNN architecture in the form of a feature extractor as shown in Figure 3. The experimentations performed through the utilization of CNN model has been considered a baseline model for extracting the features from a particular MRI slice or full brain volume by passing it through the network of 2D and 3D, respectively, as shown in Figure 4. Firstly, a 2D CNN network architecture using the 2D convolutions was deployed, on the extracted slices (2D images) from the full brain volume MRI scans after the conversion from NiFti to PNG format and outputs were subject classes as CN, MCI, and AD. As the images being converted are of small and nearly moderate size, therefore, the filter size of (3 × 3) has been employed and later the max-pooling the parameters have been experimented using (2 × 2) filter sizes with stride size of 1. Likewise, it is clear observation that the larger the size of filter and strides help in shrinking a large image to such an extent and then go back with the convention stated for the architecture being deployed. Further, network architecture comprises 4 blocks of convolution layers and a rectified linear unit (ReLu), followed by 2 fully connected layers (dense layer), mapping the output of last block to output layer.

However, the issues with 2D CNN are in selecting the best slice or slices and their orientation as training inputs for the network. Thus, the recommendation is the “appropriate scan” or “best multiple slices” for efficient results, which somewhat obscures the slice selection criteria. Any time, this is problematic and impractical. Thus, the concentration on the few scans and orientations around the image can lose out the crucial details as well as features required for the efficient deployment of CNN architecture. So the easiest and simplest way to ensure is to use the scans corresponding to entire brain volume, which comes with a three-dimensional pixel value, meaning a pixel value for each dimension in planar geometry extracted as (*x*, *y*, *z*). With the hypothesis that 3D CNN will perform better than 2D CNN, further 3D architecture of CNN has been developed which takes the 3D set of MRI scans as an input (NiFti format). Thus, the employed 3D architecture uses MRI volumes as a planar size with specific dimensions of 182 × 218 × 182 on the raw NiFti data. Thus, the schematic interpreted output is a single scalar value resulting adequate for the recognition of the disease. Moreover, the schematic illustration comprises of multiple repeated blocks of (3 × 3 × 3) convolution layer which has stride size of 1, a ReLU, (3 × 3 × 3) convolution layer which has stride size of 1, and max-pooling layer with stride size of 1. Likewise, the number of feature maps was set to eight in the first block and was doubled after each max-pooling layer to infer a sufficiently rich representation of the brain. The final recognition corresponding to each class is obtained by using a fully connected layer (dense layer), which maps the output of the last block to a single output value.

The article "Classification of Alzheimer's Disease Using Gaussian-Based Bayesian Parameter Optimization for Deep Convolutional LSTM Network" was retracted in 2023. Reasons: signs of a paper mill; compromised peer review; unreliable results or conclusions.

However, during the training of the machine, the user manually selects a learning algorithm and sets one or more model parameters referred to as hyperparameters before a ML model is created. It is well known that the algorithm and hyperparameters used can have a significant effect on the efficiency of the model, but their collection involves a specific knowledge and several manual iterations. Likewise, the previously developed models using both 2D and 3D CNN methods thus require the swift and determined limit for hyperparameter values to be identified in order to optimize the accuracy measurement for epochal parameters, learning rate, and optimizer. For this purpose, the methods for addition, testing, and refinement are considered along with analyses of previous research consequences to reduce the manual collection efforts corresponding to the random sample values. The process for this kind of sorting for finding best optimized model is reproduced using Algorithm 3 so that the search spaces are reduced and the parametric selection and related values are being evaluated for the whole dataset.

Finally, the application of 2D or 3D architecture for deep CNN models can be rendered to extract the features from the image that is further fed into the LSTM architecture. As shown in Figure 5, we used Conv2D and Conv3D with the addition of hidden layers that results in hybrid CNN-LSTM architecture for the extraction features followed by 2-hidden layered LSTM model mapping the output of the last block of the dense layer to an output value. We use 2 LSTM layers in which 832 cells are available for each LSTM layer and a 512-projection unit layer for dimensionality reduction. The LSTM is unrolling for 20-time phases for training with trimmed back propagation over time, unless otherwise specified back propagation through time. Moreover, a five-frame delay on the output state is further helps in easy prognosis of AD when compared with the use of current frame resulting in adequate development of framework for the detection of AD.

The article "Classification of Alzheimer's Disease Using Gaussian-Based Bayesian Parameter Optimization for Deep Convolutional LSTM Network" was retracted in 2023. Reasons: signs of a paper mill; compromised peer review; unreliable results or conclusions.

## 6. Result and Discussions

Early autodiagnosis of MCI patients at risk of progression to AD (AD vs. MCI) is more important from a therapeutic point of view than the issue of AD versus NC (AD vs. CN) for successful AD care. Since patients with late MCI are identified as having a very high chance of conversion to AD, and, more specifically, early MCI may be considered the starting point of AD, and MCI status is crucial in the early detection of AD. A correct and reliable diagnosis of MCI will lead to the identification of patients who are at a higher risk of developing dementia, as well as the provision of potential and regular care and the ability to prepare for the future. Developing a precise and effective computerized aided diagnosis method for the classification of CN, MCI, and AD patients could therefore be a significant step forward in the field of ageing science. As a result, this research carried out various experiments considering the same have been conducted and the prognosis for the AD detection through novel approach for optimal selection for detecting crucial biomarkers has been experimented.

### 6.1. Performance Evaluation

#### 6.1.1. Baseline System Using CNN Model

In this first set of experiments, an effort to evaluate for the adequate baseline system through the comparative analysis using 3D and 2D scans corresponding to both ternary (S1) and binary classification (S2, S3, and S4) has been made. It has been found that CONV-3D utilizing the 3D scans (NiFti format) has performed better with an average relative improvement of 3.19% and 3.79% in case of ternary AD vs. MCI vs.CN (S1) and binary classification models, respectively, as shown in Table 2. As expected, a 3D model framework is better at collecting spatial information in 3D volume of the neuroimages, which is important in medical images. Furthermore, the results show that typical 2D convolutional filters are incapable of detecting 2D spatial patterns and the structures, whereas 3D CNN is more capable of detecting 3D topology in MRI neuroscans, such as parahippocampal patches, temporal poles, and amygdale areas, that are directly associated with AD. In case of binary classification, the accuracy of the baseline model with AD vs. MCI (S2) subjects in the training and testing sets is observed at 73.34% which is very lower as compared to the 82.65% constituting AD vs. CN (S4)-based binary classification model. However, the clear distinction between the systems comprising AD vs. CN can be made in comparison to CN vs. MCI (S3) as it is difficult to classify the intermediate stage (i.e., MCI) from CN.

The article "Classification of Alzheimer's Disease Using Gaussian-Based Bayesian Parameter Optimization for Deep Convolutional LSTM Network" was retracted in 2023. Reasons: signs of a paper mill; compromised peer review; unreliable results or conclusions.

### 6.2. Manual Selection of Parameters Using CNN-3D Model

For parameter optimization manually and automatically, CONV-3D models (S1 to S4) are carried forward based on their best performance out of 2D and 3D CNN.

#### 6.2.1. Performance Evaluation on Varying Learning Rates

In this first set for parameter optimization, the learning rate varying at 0.0010 to 0.0030 for the four abovementioned systems S1, S2, S3, and S4 has been experimented. The varying of the learning rate at the end of each batch helps in the adequate monitoring of weight and dynamics; thus, one can make for the conclusion for the influence on the corresponding weight update. The result showcases the better performance at 0.0025 learning rate in case of ternary system S1, whereas 0.0020 for all the three binary systems S2, S3, and S4 as detailed in Table 3. Likewise, there might have been different scenarios given for the inclusion of other parameters leading to wide range of permutation selections across the hyperparameters. Given on the case of manual selection, systems S1, S2, S3, and S4 have resulted in 3.63%,3.83%, 1.61%, and 2.04% of RI, respectively. Best models S1 with a learning rate of 0.0025 and S2, S3, and S4 with 0.0020 are further carried forward for next-level hyperparameter optimization.

#### 6.2.2. Performance Evaluation on Varying Optimizers

The other important selection is the use of algorithms or methods helpful in changing the attributes of utilized neural network such as weights and learning rate with an objective of reducing the losses. The four different optimizers including SGD, RMSprop, Adam, and Adamax have been experimented in Table 4 based upon their best learning rate as obtained in Table 3. For system S1, the Adam optimizer with learning rate 0.0025, no change has been observed for the ternary system of classification. Likewise, for the case of binary classification system with learning rate of 0.0020, Adamax in S2 and S4 and RMSprop in S3 has led to the RI of 3.92%, 2.91%, and 1.04% for the given architecture of 3D-based convolutional network. The models which obtained the highest accuracy with respect to different optimizers are moved to next-level hyperparameters tuning.

The article "Classification of Alzheimer's Disease Using Gaussian-Based Bayesian Parameter Optimization for Deep Convolutional LSTM Network" was retracted in 2023. Reasons: signs of a paper mill; compromised peer review; unreliable results or conclusions.

#### 6.2.3. Performance Evaluation on Varying Hidden Units

Further parametric optimization experiments have been performed on the hidden units which have been considered an additional object in the scope of such classification learning. Likewise, the four systems S1, S2, S3, and S4 with the use of preselection of their respective learning rates and optimizers from Tables 3 and 4 have been further varied with the hidden units varying as [64, 128, 256, 512] in Table 5 for better utilization of the affine transformation through the use of elementwise nonlinear functionality. Thus, the results have concluded to the use of 256 hidden units for S1, 512 for S2 and S3, likewise, 128 hidden units for the S4 model. The difference outlined in the set of binary classification is clearly based on the availability for the number of subjects as well as scans corresponding to particular subject.

Finally, for the manual selection of the parameters, the observations as detailed in Table 6 corresponding to both ternary system (S1) and binary systems (S1, S2, S3, and S4) alongside their RI in comparison to the baseline 3D CNN architecture in Table 2 has been obtained.

### 6.3. For Proposed Automatic Selection of Parameters Using CNN-3D Model

The tuning of hypermeters for the abovementioned systems S1, S2, S3, and S4 (CONV-3D) has been done by the means of Bayesian optimization such that the automatic selection will help in reduction of the time spent and even result in better generalisation on the corresponding testing dataset. The process as detailed in Algorithm 3 has been taken into account for getting the two best hyperparameter combination schemes being represented as BOS-1 and BOS-2. The approach likewise has used a smaller number of iterations in comparison to traditional and manual selection approaches, and likewise, the training for the model is limited as they expected to generate a highest validation score in the earlier provided settings.  Table 7 showcases the performance of automatically fetched hyperparameter models for the four systems which is quite different in comparison to the manual selection where the choice of first selection remained anomalous. Therefore, the relative improvement of 2.73% for S2 and 5.15% for S3 has been obtained for the best model scheme selection (BOS-1) in comparison to the manual selection of parameters done in Table 6. And no changes have been noticed for models S1 and S4.

The article "Classification of Alzheimer's Disease Using Gaussian-Based Bayesian Parameter Optimization for Deep Convolutional LSTM Network" was retracted in 2023. Reasons: signs of a paper mill; compromised peer review; unreliable results or conclusions.

### 6.4. Performance Evaluation through Augmentation for Obtained Optimized Model Using LSTM

Finally, the experiments using rotational process of image augmentation has been performed which has served to be a handy strategy for synthetically increasing the size of the training set without having a need to acquire new images while performing experiments on CNNs. Based on the results obtained from Table 7, the best model (BOS-1) has been selected and the original data has been replicated with synthesised photos employing slighter variations, LSTM has been employed with CNN-3D architecture so that with the presence of dense images, the model is well able to learn from such augmented examples with results as detailed in Table 8. Further, it can be observed that the fusion of original, 180-degree and 270-degree rotational datasets has outperformed individual rotational metric. Therefore, the RI of 2.42%, 2.13%, 3.33%, and 3.79% for systems S1, S2, S3, and S4 have been obtained.

### 6.5. Comparative Analysis of Proposed Method with Earlier Approaches for AD Detection

Earlier techniques utilized by researchers obtained precision somewhere in identifying individuals with normal control subjects by different datasets of Alzheimer's disease. It is completely obvious that the intermediary stage between CN and AD is MCI and that this stage is the most difficult to identify. Also, a relatively limited number of research have finally taken account of the MCI group [64], and, given this procedure, very little effort has been made to choose parameters appropriately. This section contains a comparison study of the proposed methodology with prior state-of-the-art strategies for appropriate AD categorization. The study, as shown in Table 9, portrays the use of multiple datasets and multimodality testing, which results in both hypotheses, and such detailed analysis helps the community in enhancing the general data levels as well as specified occasions for the objective of parameterisation during model training.

## 7. Conclusion

An early detection of AD allows the patient to receive the best therapeutic conceivable. Numerous researchers are working on this difficult problem, and many approaches for diagnosing AD have already been created. In this work, we first trained, validated, and evaluated 2D and 3D CNN on the ADNI MRI dataset and conducted binary classification such as AD-MCI, AD-CN, and MCI-CN, as well as multiclass ternary classification involving AD-MCI-CN. As a result, the best model out of 2D and 3D CNN was carried forward for optimization based on the both manual selection and automatic selection of hyperparameters including learning rate, optimizers, and dense units by Bayesian optimization was developed. Furthermore, on the Bayesian optimized 3D CNN model, we developed a pooled hybrid CNN-LSTM technique to identify the prognosis of AD disease employing data augmentation in our proposed process. In comparison to traditional and manual selection procedures, the strategy has utilized fewer iterations, and the training for the model has also been constrained, since they aim to provide the greatest validation score in the previously stated conditions. Therefore, an overall relative improvement of 7.03%, 12.19%, 10.80%, and 11.99% was achieved, in which the best model is obtained for systems S1, S2, S3, and S4. The study can be expanded over in the future by incorporating different other frameworks, such as VGG16, VGG19, AlexNet, and DenseNet. In addition to the proper use of the transfer learning for effective AD projections, the proposed methodology for Gaussian-based Bayesian optimization of parameters can be applied. Moreover, we focused only on MRI modality in our work; in the future, this work could be expanded with the inclusion of other modalities like PET, DTI, and fMRI scans.

The article "Classification of Alzheimer's Disease Using Gaussian-Based Bayesian Parameter Optimization for Deep Convolutional LSTM Network" was retracted in 2023. Reasons: signs of a paper mill; compromised peer review; unreliable results or conclusions.

## Figures and Tables

**Figure 1:** Extracted slices of CN, MCI, and AD patients MRI scans from (a) to (c), respectively.

**Figure 2:** Visualization for no. of patients against CDR score.

**Figure 3:** CNN architecture for prognosis of AD.

**Figure 4:** Block diagram of baseline system for AD classification using 2D and 3D convolution network.

**Figure 5:** Block diagram for AD classification using deep convolution LSTM network.

**Algorithm 1:** Dataset preprocessing.

**Algorithm 2:** Increasing the size of dataset with rotation with an angle 180 or 270 degrees.

**Algorithm 3:** Optimal selection of hyperparameter using Gaussian-based Bayesian parameter optimization for AD classification.

**Table 1:** Demographic Information constituting MRI scans of cohorts.

Subjects/cohorts	Number of males	Number of females	Age range	Avg. age	Avg. CDR score
CN	97	106	56-95	77	0.109
MCI	30	23	62-91	79	0.75
AD	61	48	56-89	75	1

**Table 2:** CONV-2D and CONV-3D performance comparative evaluation binary/ternary for AD classification.

Dataset		System type	Accuracy (%)	
Training set	Testing set		CONV-2D	CONV-3D
AD, MCI, CN	AD, MCI, CN	S1	71.59	73.96
AD, MCI	AD, MCI	S2	69.47	73.34
CN, MCI	CN, MCI	S3	73.05	75.02
AD, CN	AD, CN	S4	79.91	82.65

**Table 3:** Impact on validating learning rate on four systems using CONV-3D network architecture.

Learning rate	Accuracy (%)			
	S1	S2	S3	S4
0.0010	71.65	70.56	74.56	81.87
0.0015	73.96	73.34	75.02	82.65
0.0020	75.18	76.15	76.23	84.34
0.0025	76.65	74.87	75.97	83.56
0.0030	74.36	74.96	75.56	82.54

The article "Classification of Alzheimer's Disease Using Gaussian-Based Bayesian Parameter Optimization for Deep Convolutional LSTM Network" was retracted in 2023. Reasons: signs of a paper mill; compromised peer review; unreliable results or conclusions.

**Table 4:** Impact on validating optimizers on four systems using CONV-3D network architecture.

Optimizer	Accuracy (%)			
	S1	S2	S3	S4
SGD	73.65	70.52	70.69	80.24
RMSprop	74.85	72.54	77.21	82.89
Adam	76.65	76.15	76.23	84.34
Adamax	75.15	76.86	74.64	85.22

**Table 5:** Impact on validating hidden units on four systems using CONV-3D network architecture.

#units	Accuracy (%)			
	S1	S2	S3	S4
64	73.96	74.56	73.86	82.40
128	74.85	75.43	75.56	86.28
256	76.65	76.15	77.21	85.22
512	75.59	76.99	77.56	85.84

**Table 6:** Observational performance evaluation on manual selection of parameters for CONV-3D architecture.

System	Parameters	Accuracy(%)
S1	Lr = 0.0025; opt = Adam; hidden_units = 256	76.65
S2	Lr = 0.0020; opt = Adamax; hidden_units = 512	76.99
S3	Lr = 0.0020; opt = RMSprop; hidden_units = 512	77.56
S4	Lr = 0.0020; opt = Adamax; hidden_units = 128	86.28

**Table 7:** Accuracy of CONV-3D on four systems using Bayesian optimization for optimal selection of parameters.

Model type	System	Parameters	Accuracy (%)
BOS-I	S1	Lr = 0.0025; opt = Adam; hidden_units = 256	76.65
	S2	Lr = 0.0015; opt = MSprop; hidden_units = 128	78.23
	S3	Lr = 0.0020; opt = Adam; hidden_units = 128	77.96
	S4	Lr = 0.0020; opt = Adamax; hidden_units = 128	86.28

BOS-2	S1	Lr = 0.0020; opt = Adamax; hidden_units = 256	75.78
	S2	Lr = 0.0020; opt = Adam; hidden_units = 128	77.19
	S3	Lr = 0.0020; opt = Adamax; hidden_units = 128	76.65
	S4	Lr = 0.0020; opt = Adamax; hidden_units = 128	85.95

**Table 8:** Accuracy obtained on augmented ternary and binary classification systems employing hybrid CNN-LSTM architecture.

Model type	Augmentation type	Accuracy (%)			
		S1	S2	S3	S4
BOS-I	None	77.29	80.56	80.44	89.18
	180	77.93	80.81	81.04	90.64
	270	77.90	80.84	80.23	90.46
	180 + 270	79.16	82.28	83.12	92.56

**Table 9:** Comparative analysis of AD classification system using earlier proposed techniques.

Author name (year)	Dataset details	Methods and approaches	Summary
Li et al. [65] (2020)	ADNI-1 including MRI as well as PET brain scans	LDF-based modelling predicated on the combination of low-ranking and discriminant correlations representation through fusion of multimodal datasets	The researcher experimented for the adequate extraction of latent characteristics for submodal data using the low-level representation approach which has helped in removing noise information and an enhanced system performance
El-Sappagh et al. [66] (2020)	MRI brain scans	A multitasking deep learning framework based on the five series data paradigms towards Alzheimer progression and detection on fused CNN-BiLSTM	The authors demonstrated a model that predicts AD progression as a multiclass classification task and four critical cognitive scores as regression tasks. The experimental results have shown the model to be medically advanced
Suárez-Araujo et al. [67] (2021)	ADNI dataset consisting with sample of 128 MCI patients and 203 controls.	A hybrid ANN-based AD classification system	The ANN method suggested achieves good diagnosis accuracy, even if it is just based on conventional medical trials. These findings indicate that method is particularly appropriate for primary treatment, helping doctors to work with suspicion of cognitive impairment
Pei et al. [68] (2021)	ADNI	Pseudo-3D block and an enlarged global context block, incorporated in a cascaded approach utilizing long-range dependencies into the a remnant backbone block	Experimental findings done by the authors show 89.27% of the AD/NC accuracy and 87.57% of the light cognitive impairments/NC with CNN modelling while 0.5% more accurate than the backbone is reported
Tomassini et al. [69] (2021)	ADNI and OASIS	3D-ConvLSTM-based early AD diagnosis mechanism utilizing full-resolution brain images	The researcher proposed a framework which works effectively to distinguish between CN and AD patients with a classification accuracy of 86% conducted using a modular GPU cloud service
Proposed approach	ADNI	Bayesian optimization with binary as well as ternary classification on augmented 3D-MRI data scans employing long short-term memory (LSTM)	The method used fewer iterations, and the model training was improved alongside obtaining the highest validation score on both ternary as well as binary classification

The article "Classification of Alzheimer's Disease Using Gaussian-Based Bayesian Parameter Optimization for Deep Convolutional LSTM Network" was retracted in 2023. Reasons: signs of a paper mill; compromised peer review; unreliable results or conclusions.

## Data Availability

The data that support the findings of this investigation are available from ADNI (http://adni.loni.usc.edu); however, they are subject to restrictions because they were utilized under permissions for this work and are therefore not publicly available. The authors' data are, however, available upon reasonable request and with ADNI's approval.
